The article "Unveiling the Nexus: Influence of learning motivation on organizational performance and innovative climate of Chinese firms" was retracted in 2024. Reasons: unreliable data; unreliable results or conclusions; concerns about the data; concerns about the results or conclusions.

# Unveiling the Nexus: Influence of learning motivation on organizational performance and innovative climate of Chinese firms

**DOI:** 10.1371/journal.pone.0304729

**Published:** 2024-05-31

**Authors:** Yu Zhang, Caizhi Liao, Jialei Liu, Yihe Zhang, Shiquan Gui, Qing Wei

**Affiliations:** 1 Development and Planning Division, Chengdu University, Chengdu, Sichuan, China; 2 School of Continuing Education, Chengdu University, Chengdu, Sichuan, China; University of Central Punjab, PAKISTAN

## Abstract

This study delves into the interplay between learning motivation, organizational performance, and the innovative climate within Chinese firms. It is a subject of frequent discussion in literature but there is little concrete evidence supporting this viewpoint within the context of small and medium size enterprises in China. Drawing upon a comprehensive review of existing literature and empirical data gathered, this research aims to uncover the connections between employee learning motivation and its impact on the organizational dynamics in the context of Chinese firms. A cross sectional survey is used to collect the data of 115 Chinese firms and structural equation modelling (SEM) is used for empirical analysis. The results show that success of firms in terms of innovation is significantly influenced by organizational learning motivation. Moreover, innovative environment of the firms increases the overall performance of the organizations. It is also found that factors affecting the innovations have a significant impact on organizational performance. The findings of the study suggest that firms should develop organizational learning motivation to boost their innovation capability and overall performance. This study offers insights and recommendations for organizations and policymakers seeking to harness the potential of learning motivation to drive sustainable growth, competitiveness, and innovation in Chinese firms.

## 1. Introduction

The learning motivation of an organization can be defined as "a field toward to the study of cognitive and social processes of knowledge in organizations that are imbricated in organizational and work practices" [1]. It refers to the drive, desire, or willingness of individuals within an organization to engage in learning activities, acquire new knowledge, develop skills, and improve performance within the organizational context [2, 3]. Organizational learning motivation is crucial as it directly impacts the willingness of employees to engage in learning activities, acquire new knowledge, and apply these skills to enhance individual and collective performance [4, 5]. Organizations can maximize their competitive advantage by placing a high priority on learning in such settings [6]. Organizational learning is essential for enabling organizations to produce, distribute, and integrate knowledge and experience while promoting continual learning. The organizational characteristics that encourage learnings are included in the capacity for organizational learning [7]. This capability includes all organizational and administrative practices that aid in learning [4]. It is a collection of procedures that improve capacity of an organization to sustain and improve performances or a set of operational procedures that promotes learning [8].

The article "Unveiling the Nexus: Influence of learning motivation on organizational performance and innovative climate of Chinese firms" was retracted in 2024. Reasons: unreliable data; unreliable results or conclusions; concerns about the data; concerns about the results or conclusions.

There is an established relationship in the literature, between organizational learning and organizational performance. Organizational performance is the measure of how effectively an organization achieves its objectives and goals. It encompasses various aspects of an organization’s functioning, including its efficiency, productivity, profitability, quality of products or services, customer satisfaction, innovation, and overall success in meeting stakeholder expectations [9]. Key components that contribute to assessing organizational performance include metrics such as revenue growth, profitability, return on investment, and cost efficiency [10]. Assessing the morale, motivation, and commitment of employees, which can significantly impact productivity, innovation, and overall organizational success [4, 6].

Innovative climate in firms is also an aspect that affects the learning motivation and organizational performance of the firms. The innovative climate of a firm includes the environment, culture, and conditions within an organization that foster and encourage creativity, experimentation, and the development of new ideas, products, processes, or services [11]. It is the collective mindset, values, practices, and structures that shape how innovation is perceived, supported, and implemented across the organization [12]. An innovative climate thrives on a culture that encourages creative thinking, where employees feel empowered to share ideas without fear of criticism. It also embraces calculated risk-taking, understanding that not all innovations will succeed but valuing the lessons learned from experimentation [7]. An environment that promotes open communication, collaboration, and cross-functional teamwork fosters the exchange of ideas and perspectives. This diversity of thought often leads to more innovative solutions to challenges. A culture that values learning and ongoing development nurtures an environment where employees are encouraged to explore new skills, knowledge, and trends [12, 13].

The relationship among organizational learning motivation, innovative climate, and the performance of firms is complex and interconnected. Organizational learning motivation is a key driver of an innovative climate [14]. When employees are motivated to learn and develop their skills, they are more likely to come up with new ideas, embrace change, and contribute to the organization’s innovation culture [8]. An organization that promotes learning motivation creates an environment where employees feel encouraged to take risks, experiment, and think creatively, which are crucial elements of an innovative climate [15]. On the other side, an innovative climate is positively associated with the performance of firms. When an organization fosters a culture of innovation, it tends to develop new products or services that meet customer needs, gain a competitive advantage, improve processes and operations, leading to increased efficiency [5]. Organizational learning motivation leads to an innovative climate, which, in turn, enhances the performance of firms [10]. Higher performance can further motivate employees to learn, innovate, and maintain a positive innovative climate [8]. As the organization’s performance improves, it can invest in resources, training, and tools that promote learning and innovation, further strengthening the cycle [11–16].

The article "Unveiling the Nexus: Influence of learning motivation on organizational performance and innovative climate of Chinese firms" was retracted in 2024. Reasons: unreliable data; unreliable results or conclusions; concerns about the data; concerns about the results or conclusions.

There is extensive literature on this topic but there are still several unanswered questions that warrant further investigation. While it is known that learning motivation influences organizational performance and innovative climate, the specific mechanisms through which this occurs remain unclear. Further research is needed to identify the factors that may enhance or inhibit the relationship between learning motivation and organizational outcomes like experimentation, risk, interaction, and dialogue. Despite the theoretical advances, there is a need for research that translates findings into actionable strategies and best practices for Chinese firms. It means that while there is existing theoretical knowledge about topics like learning motivation and organizational performance, there is a gap in translating this knowledge into practical, implementable strategies for Chinese firms. This translation is necessary because theoretical knowledge, while valuable, may not always directly translate into effective actions or practices that can be applied in real-world business settings. To achieve this translation requires several steps like understanding the context. Researchers need to understand the specific context of Chinese firms, including cultural, economic, and regulatory factors that may impact the applicability of theoretical findings. Then there is need to identify the key challenges faced by Chinese firms in implementing theoretical concepts and develop strategies that specifically address these challenges. Based on theoretical insights and empirical evidence, researchers can develop actionable recommendations and best practices that are tailored to the unique needs and circumstances of Chinese firms. Finally, these actionable strategies and best practices should be disseminated to Chinese firms through channels such as academic journals, conferences, and industry publications, and efforts should be made to facilitate their implementation through training programs and consulting services.

The article "Unveiling the Nexus: Influence of learning motivation on organizational performance and innovative climate of Chinese firms" was retracted in 2024. Reasons: unreliable data; unreliable results or conclusions; concerns about the data; concerns about the results or conclusions.

Studies that explore the practical implications of enhancing learning motivation for organizational performance and innovation management can provide valuable guidance for managers and policymakers [17, 18]. Addressing these unanswered questions can lead to more effective strategies for fostering learning, innovation, and sustainable growth. The problem addressed in the research paper likely focuses on understanding the relationship between learning motivation, organizational performance, and innovative climate within Chinese firms. The study aims to explore how learning motivation among employees influences overall organizational performance and examines how motivated employees contribute to achieving organizational goals and objectives. Another aspect is examining the role of learning motivation in fostering an innovative climate. This involves assessing the impact of motivated employees on creativity, idea generation, knowledge sharing, and the implementation of innovative practices and technologies. The paper also discusses the practical implications of its findings for Chinese firms aimed at enhancing learning motivation and fostering a culture of innovation. This study can provide insights into how to cultivate a culture that encourages creativity, experimentation, and the adoption of new ideas and technologies. Research in this area can contribute to the theoretical understanding of organizational learning motivation, organizational performance and innovative climate. Overall, this study provides valuable insights that can inform both academic theory and practical strategies for organizational development and success in today’s competitive global marketplace.

The research problem of the study could be formulated as that despite the acknowledged importance of organizational learning and innovation for sustained competitive advantage, there remains a gap in understanding how individual learning motivation influences organizational performance and the innovative climate within Chinese firms. The research gap in the study likely revolves around the specific challenges faced by Chinese organizations in fostering and maintaining high levels of learning motivation among their employees. Chinese organizations may face challenges in aligning their organizational culture with a culture that promotes learning and innovation. Traditional Chinese culture values stability and conformity, which may inhibit risk-taking and innovation. The effectiveness of learning motivation strategies may be impacted by the quality and nature of China’s educational system. Issues such as rote learning and exam-focused education could hinder employees’ intrinsic motivation to learn and innovate. Moreover, Chinese organizations may struggle with leadership styles that do not encourage or support a culture of learning and innovation. Autocratic leadership, which is common in Chinese organizations, may stifle creativity and risk-taking. Limited resources, both financial and human, could pose challenges for Chinese organizations in implementing effective learning motivation strategies. This could include constraints on training budgets, lack of access to learning opportunities, or insufficient time for employees to engage in learning activities. In addition, the pace of technological change in China may require employees to continuously learn new skills and adapt to new technologies. Organizations that fail to facilitate this ongoing learning process may struggle to maintain a competitive edge and with increasing globalization, Chinese organizations are facing greater competition from international firms. This places pressure on organizations to innovate and adapt quickly, which may require a high level of learning motivation among employees. This study seeks to address this gap by examining the relationship between learning motivation, organizational performance, and the innovative climate in Chinese firms. Moreover, the significance of the study lies in its potential to contribute to both theory and practice in several ways. This study provides valuable insights into the role of learning motivation in driving organizational performance and fostering an innovative climate, particularly within the context of Chinese firms. This can help advance theoretical understanding of the mechanisms through which individual motivation impacts organizational outcomes. By focusing on Chinese firms, the findings offer practical implications for managers and policymakers in Chinese firms, providing them with evidence-based strategies to enhance learning motivation among employees, improve organizational performance, and promote a more innovative climate. Finally, the study adds to the growing body of literature on organizational learning and innovation, offering new perspectives and insights that can stimulate further research in this important area.

The article "Unveiling the Nexus: Influence of learning motivation on organizational performance and innovative climate of Chinese firms" was retracted in 2024. Reasons: unreliable data; unreliable results or conclusions; concerns about the data; concerns about the results or conclusions.

This study has the objective to explore the impact organizational learning motivation including its aspects experimentations, risk, interaction, and dialogue that are most effective in different organizational contexts and these are little focused in the earlier literature related to Chinese firms. Extending this finding would explore the ways in which learning motivation influences the organizational performance. Moreover, this study also has the objective to consider the impact of aspects of innovation performance like efficiency and efficacy on performance of Chinese firms by collecting the primary data and applying the econometric techniques for empirical analysis. It is found that learning motivation of employees positively influences the innovations and performance of workers in Chinese firms.

## 2. Theoretical foundations

The theoretical relationship among organizational learning motivation, innovation capacity and organizational performance is grounded in several perspectives. Social learning theory posits that individuals learn through observation, imitation, and social interaction. Within organizations, employees’ learning motivations can be influenced by observing the behaviors and outcomes of others. When employees witness colleagues being rewarded or recognized for their learning efforts, they are more likely to be motivated to engage in similar learning activities. This social reinforcement of learning motivation contributes to improved individual and organizational performance [19]. Expectancy theory suggests that individuals are motivated to engage in behaviors when they believe that their efforts will lead to desired outcomes. In the context of organizational learning, employees who are motivated to learn are more likely to believe that their learning efforts will result in improved job performance, career advancement, and personal development. This belief in the expectancy of positive outcomes drives employees to invest time and effort in learning activities, ultimately enhancing organizational performance [20]. Goal setting theory emphasizes the importance of setting specific, challenging goals to motivate individuals and improve performance. Organizational learning motivation can be facilitated by setting clear learning goals and providing employees with the necessary resources and support to achieve them. When employees are motivated to attain these learning goals, they are more likely to acquire new knowledge and skills that contribute to enhanced job performance and organizational effectiveness [21]. Self-determination theory proposes that individuals are intrinsically motivated to pursue activities that fulfill their psychological needs for autonomy, competence, and relatedness. In the context of organizational learning, employees are more likely to be motivated when they have opportunities to autonomously choose learning activities that align with their interests and goals, when they feel competent in their ability to learn and apply new knowledge, and when they experience a sense of connection and belongingness within the organization. Meeting these psychological needs for motivation fosters a positive learning environment and leads to improved organizational performance [22]. The resource-based view of the firm suggests that organizational learning capabilities, including the motivation of employees to learn and adapt, are a source of competitive advantage. Organizations that invest in fostering a learning culture and motivating employees to continuously improve their knowledge and skills are better positioned to adapt to changing market [23]. The knowledge-based view emphasizes the role of knowledge creation, sharing, and utilization as critical drivers of organizational innovation. Organizational learning motivations facilitate the acquisition and development of new knowledge and skills among employees, which are essential for generating innovative ideas, processes, and products. As employees engage in learning activities and accumulate knowledge, they are better equipped to identify opportunities for innovation and contribute to the organization’s overall innovation capacity [24]. Learning organization theory suggests that organizations capable of continuously learning and adapting are more likely to innovate and achieve long-term success. Organizational learning motivations play a central role in cultivating a learning-oriented culture and mindset within the organization, where employees are encouraged to experiment, take risks, and learn from both successes and failures. This culture of learning fosters an environment conducive to innovation, where employees feel empowered to generate and implement novel ideas to address organizational challenges and opportunities [11]. Innovation diffusion theory highlights the importance of individual and organizational learning processes in the adoption and implementation of innovations. Organizational learning motivations drive the dissemination of new knowledge and best practices throughout the organization, facilitating the adoption of innovative ideas and technologies. As employees become motivated to learn and apply new knowledge, they become champions and advocates for innovation within their respective teams and departments, leading to widespread adoption and integration of innovative practices across the organization [25]. Absorptive capacity theory suggests that organizations must have the ability to recognize, assimilate, and apply external knowledge to innovate effectively. Organizational learning motivations contribute to the development of absorptive capacity by enhancing employees’ skills in identifying relevant external knowledge sources, evaluating the quality and applicability of incoming information, and integrating new knowledge into existing organizational routines and processes. By fostering a culture of continuous learning and knowledge exchange, organizations can enhance their absorptive capacity and leverage external knowledge to drive innovation [26]. The Triple Helix model posits that innovation is driven by interactions between academia, industry, and government. Organizational performance is enhanced when these stakeholders collaborate effectively to create and transfer knowledge, develop new technologies, and stimulate economic growth. Innovation capacity serves as a catalyst for collaboration within the Triple Helix framework, as organizations with strong innovation capacities are better positioned to leverage external knowledge and expertise, forge strategic partnerships, and participate in collaborative innovation ecosystems, ultimately leading to improved performance outcomes [27].

The article "Unveiling the Nexus: Influence of learning motivation on organizational performance and innovative climate of Chinese firms" was retracted in 2024. Reasons: unreliable data; unreliable results or conclusions; concerns about the data; concerns about the results or conclusions.

## 3. Conceptual framework

A conceptual framework outlining the relationship among organizational learning motivation, innovation capacity and organizational performance can be structured as shown in the following Fig 1. At the individual level, the study considers the concept of learning motivation, which is influenced by different factors while learning motivation is expected to drive individual learning behavior and the acquisition of new knowledge and skills. At the organizational level, the study focuses on two key outcomes: organizational performance and the innovative climate. Organizational performance is a multifaceted construct that includes financial performance, operational efficiency, and overall effectiveness. The innovative climate refers to the organizational culture and practices that support and encourage innovation among employees. The study also proposes that individual learning motivation can influence organizational performance and the innovative climate through mediating mechanisms. Resource-Based view theory suggests that a firm’s unique resources and capabilities are key drivers of competitive advantage and, consequently, organizational performance. According to this theory, firms with valuable, rare, and difficult-to-imitate resources are more likely to outperform competitors. Moreover, agency theory examines the relationship between principals (e.g., shareholders) and agents (e.g., managers) in an organization. It suggests that conflicts of interest between principals and agents can impact organizational performance. For example, managers may prioritize their own interests over those of shareholders, leading to suboptimal performance. The Fig 1 highlights the conceptual framework of the study.

The article "Unveiling the Nexus: Influence of learning motivation on organizational performance and innovative climate of Chinese firms" was retracted in 2024. Reasons: unreliable data; unreliable results or conclusions; concerns about the data; concerns about the results or conclusions.

**Fig 1:** Conceptual framework. https://docs.google.com/document/d/1QNspQeJBQQDAaH8VKCbQbj_KLjl_syej/edit?usp=sharing&ouid=109167264099591876564&rtpof=true&sd=true.

Organizational learning motivation refers to the collective drive and willingness of individuals within an organization to engage in learning activities, acquire new knowledge, and develop skills that contribute to personal and organizational growth. When employees are motivated to learn and grow, they are more likely to be engaged in their work, resulting in higher levels of commitment, productivity, and job satisfaction [28]. Engaged employees are also more inclined to contribute discretionary effort, proactively seek opportunities for improvement, and collaborate effectively with colleagues, all of which contribute to improved organizational performance. Organizational learning motivation also drives employees to actively seek out new information, engage in training and development initiatives, and apply their learning to solve problems, innovate, and make informed decisions [29]. The acquisition and application of relevant knowledge and skills enhance employees’ capabilities, performance, and contributions to organizational goals. When employees are motivated to learn and develop, they contribute to the organization’s ability to achieve its strategic objectives, respond effectively to changing market conditions, and sustain competitive advantage over time [30]. Social Cognitive theory emphasizes the role of social factors in learning and motivation. According to social cognitive theory, individuals can learn by observing others (social learning) and by receiving feedback and reinforcement from others (social reinforcement). Social cognitive theory also emphasizes the role of self-efficacy beliefs in motivation, suggesting that individuals are more likely to be motivated to learn when they believe they have the ability to succeed.

Innovation capacity refers to the organization’s ability to generate, develop, and implement innovative ideas, practices, and solutions that create value for customers and stakeholders. This process contributes to the accumulation of a diverse range of knowledge and expertise within the organization, providing a rich foundation for innovation [31]. Employees who are motivated to learn are more likely to stay updated with industry trends, emerging technologies, and best practices, thereby fueling the organization’s ability to generate innovative ideas and solutions. Motivated learners are more inclined to engage in creative thinking and problem-solving activities. By fostering a culture of experimentation, curiosity, and risk-taking, organizational learning motivation encourages employees to explore new possibilities, challenge conventional wisdom, and think outside the box [32]. This creative mindset is essential for generating novel ideas, designs, and approaches that drive innovation and address complex challenges faced by the organization. Moreover, organizational learning motivation enhances the organization’s adaptability and flexibility in response to changing market conditions, customer preferences, and competitive pressures [33]. Motivated employees are more willing to embrace change, adapt to new technologies and methodologies, and experiment with alternative approaches to problem-solving. This adaptability enables the organization to continuously evolve and adjust its strategies, processes, and products in line with emerging opportunities and threats, thereby maintaining a competitive edge in the marketplace [34]. Learning-motivated employees are more likely to collaborate with colleagues from diverse backgrounds, departments, and disciplines. By sharing knowledge, exchanging ideas, and leveraging each other’s strengths and expertise, employees can generate synergies and cross-pollinate insights that stimulate innovation [35]. Collaborative learning environments foster creativity, spark new perspectives, and facilitate the co-creation of innovative solutions that draw upon a wide range of perspectives and expertise within the organization. Diffusion of Innovation theory explains how innovations spread within a social system. In the context of organizational climate, it suggests that an organization’s climate can either facilitate or inhibit the adoption and implementation of new ideas and practices. While complexity theory views organizations as complex adaptive systems that constantly evolve and adapt to their environment. In this view, an innovative climate emerges from the interactions between individuals, teams, and the larger organizational system. Moreover, creative problem solving theory focuses on the cognitive processes involved in generating creative solutions to problems. An innovative climate provides the conditions necessary for individuals to engage in creative problem-solving, such as autonomy, resources, and support from others. In addition, organizational learning theory emphasizes the importance of continuous learning and adaptation for organizational success. An innovative climate fosters organizational learning by encouraging experimentation and reflection on outcomes.

The article "Unveiling the Nexus: Influence of learning motivation on organizational performance and innovative climate of Chinese firms" was retracted in 2024. Reasons: unreliable data; unreliable results or conclusions; concerns about the data; concerns about the results or conclusions.

### 3.1. Literature review and hypotheses

The learning aptitude of the organization defined as "the ability of an organization to process knowledge, i.e., the ability to create, acquire, transfer and integrate knowledge and, also, to modify the behavior to reflect the new cognitive situation, with the aim at improving organizational performance" [16]. The idea of learning competency of organization, that includes both real and vague resources as well as aptitudes that support reasonable advantage, acts as a catalyst in organizational learning process [17]. This in turn helps the organizational learning process to advance [18]. While organizational learning ability refers to the organization’s power to fascinate and alter new information before using it to quickly produce innovative goods that have a competitive advantage [19]. In addition, aptitude for learning ability of organization functions as together an intrinsic administrative characteristic and a managerial attribute [7]. Furthermore, apart from its role in easing the learning process within organizations, it actively contributes to the learning process itself and characterize it as the removal of limitations or impediments within the organizational learning process [20, 35].

To encourage creation of organizational awareness, organizations should set up procedures and enact policies. These processes include internalization, socialization, and externalization along with variety of management techniques that support a learning environment [8]. “These practices are the foundation of organizational learning capability, which can be characterized as a set of management practices that facilitate the learning process or as a set of mechanisms that improve the organization’s ability to sustain and improve its performance” [8, 18].

The characteristics that support organizational learning were examined by earlier studies [7]. In order to achieve this, they created a scale that had five dimensions: The aspects include a propensity for risk, engagement with the outside world, conversation, and collaborative decision-making. The scale has furthermore been used in earlier investigations [6, 8, 20–22] and this study likewise makes use of these scales. Experimentation refers to how much fresh ideas and recommendations are accepted and managed within the business [6]. It is associated with endorsing novel concepts, offering positive feedback to employee initiatives, and fostering and facilitating change. Additionally, it includes looking for imaginative answers to difficulties that are based on the prospective use of various techniques and processes. One way to institutionalize organizational learning within the organization is through experimentation [5, 36].

The article "Unveiling the Nexus: Influence of learning motivation on organizational performance and innovative climate of Chinese firms" was retracted in 2024. Reasons: unreliable data; unreliable results or conclusions; concerns about the data; concerns about the results or conclusions.

Competition, social and economic systems, and policies are only a few examples of the external environment that a company interacts with. These elements have an impact on the business but are beyond of its direct control. This dimension includes metrics related to information exchange and employee involvement with the outside world, as well as the collection and transmission of external environmental data [7]. The transmission of knowledge, the development of skills, and active engagement in internal problem-solving are the three ways that learning occurs in uncertain contexts [23]. The level of tolerance an organization has for ambiguity, uncertainty, and mistakes determines its propensity to take risks. Organizations that see inaccuracies as intolerable do not foster learning, as prospective blunders may in fact promote learning. the ability to take chances without endangering the company and the willingness to face new challenges are all indicators of a person’s propensity to take risks [7, 23, 24]. An organization can apply modifications to support organizational learning, hence nurturing specific characteristics such as participative decision-making [11].

According to the literature, organizational learning and creativity frequently go side by side [25, 37]. The development of behaviors and abilities necessary for innovation is fostered by organizational learning, which is frequently seen in efforts focused on product creation [26]. Researchers that study innovation place a strong emphasis on the heroine that organizational erudition processes play in the creation of new goods. Therefore, it is clear that organizational learning is a prerequisite for any technological breakthrough [27]. Organizational learning, according to studies in this area [4, 18, 28], has a positive impact on creative performance. The first step in fostering innovation is for people to gather the most recent knowledge and then spread it throughout the company. Organizational learning and creativity are said to be closely related [19].

***H1*:** Organizational learning has a beneficial impact on organizational innovative performance.

Innovations are embraced either in reaction to shifts within internal and external contexts or as a proactive measure to shape those surroundings. SMEs are particularly well-positioned for innovation due to the inherent challenge of expanding and realizing their full capabilities [29, 37]. The essence of innovation lies in the conversion and utilization of knowledge within organizations, a process that encompasses the sharing of both knowledge and information among workforces [4, 30]. In present analysis, inventive performance is assessed through two distinct dimensions: efficacy and efficiency, a framework initially developed by the study [12]. These playwrights introduced a measurement scale for assessing artifact novelty performance, known as "innovative performance," which underwent rigorous psychometric testing and validation within the context of biotechnology firms. Efficacy seeks to evaluate the economic influence of modernization on the organization, specifically gauging the success or outcomes resulting from innovation efforts. Meanwhile, efficiency pertains to the process through which these outcomes are attained [8, 38].

The article "Unveiling the Nexus: Influence of learning motivation on organizational performance and innovative climate of Chinese firms" was retracted in 2024. Reasons: unreliable data; unreliable results or conclusions; concerns about the data; concerns about the results or conclusions.

According to earlier studies [14, 30], creative firms have the capacity to quickly adjust to environmental difficulties, leading to improved performance. Innovation improves the efficiency of SMEs [31]. The nature of the invention, the age of the organization, and the cultural context in which it functions are just a few examples of the many factors that might affect performance. The findings show that organizational learning has a stronger effect on creativity and performance in smaller firms than it does in larger ones [11, 39]. Organizational learning efforts have a greater influence on creativity in smaller organizations since there are less established organizational practices there. Using the setting of SMEs, the study [32] conducted to observe the impact of market direction, learning coordination, and modernization. According to the study’s results, learning helps to promote creativity and that advancement has a positive effect on organizational enactment. In addition, most businesses—including small and medium-sized ones, which make up a significant component of most economies—introduce new goods regularly, regardless of their level of innovation [33]. Comprehending consumer needs, monitoring competitor actions, staying attuned to technological advancements, and adhering to the principles of organizational knowledge can collectively enable organizations to harness the advantages of innovation [9]. SMEs can derive enhancements in product quality and increased sales of their manufactured products by embarking on both product innovations and market entry strategies [34]. Innovation stands as a pivotal tool for augmenting market share and conferring a competitive edge upon a company [1, 13]. This optimistic effect on a firm’s enactment culminates in an improved market position, resulting in a distinctive viable advantage and larger overall performance. Consequently, the following hypothesis is postulated:

***H2*:** Innovative performance exerts a positive impact on organizational performance.

The article "Unveiling the Nexus: Influence of learning motivation on organizational performance and innovative climate of Chinese firms" was retracted in 2024. Reasons: unreliable data; unreliable results or conclusions; concerns about the data; concerns about the results or conclusions.

Factors that promote organizational learning play a pivotal role in enhancing organizational performance in various ways. When organizations foster a culture of knowledge sharing and transfer, employees exchange information, best practices, and lessons learned [11]. This dissemination of knowledge across departments or teams enhances collective expertise, improves decision-making, and avoids redundant efforts, thus optimizing overall efficiency and performance [34, 40]. Promoting a learning culture encourages a mindset of continuous improvement. Employees are motivated to identify inefficiencies, suggest innovative solutions, and implement changes that lead to enhanced processes, better products/services, and increased productivity, ultimately contributing to improved performance metrics [35]. Organizations that prioritize learning adapt more effectively to changing environments. Employees equipped with new skills and knowledge are better prepared to navigate uncertainties, embrace change, and respond proactively to market shifts, improving the organization’s ability to stay competitive and perform well in dynamic settings [5, 36]. Learning organizations encourage creativity and innovation. By empowering employees to explore new ideas, experiment, and take calculated risks, they foster a climate conducive to innovation [21, 37]. This innovation leads to the development of new products, services, or processes that can positively impact performance by opening new market opportunities or improving operational efficiency [14, 18]. Organizations that invest in learning and development initiatives tend to have higher employee engagement and retention rates. Employees appreciate opportunities for growth, skill enhancement, and career development [24]. Engaged employees are more committed, productive, and contribute positively to organizational performance [22]. A learning-focused environment emphasizes learning from mistakes and using them as opportunities for growth. As employees acquire new knowledge and skills, they make fewer errors, make more informed decisions, and approach problem-solving more effectively, thus positively impacting overall organizational performance [9, 32]. Factors promoting organizational learning create a cycle of improvement and growth within the organization. By nurturing a culture of learning, organizations empower their employees, improve operational efficiency, foster innovation, and increase adaptability, all of which collectively contribute to improved organizational performance and sustained success.

The article "Unveiling the Nexus: Influence of learning motivation on organizational performance and innovative climate of Chinese firms" was retracted in 2024. Reasons: unreliable data; unreliable results or conclusions; concerns about the data; concerns about the results or conclusions.

***H3*:** The factors that promote organizational learning have a positive impact on organizational performance.

The organizational learning capability is made up of four parts: experimentation, propensity to risk, interaction with the external environment, and dialogue. Effective performance has features of both effectiveness and efficiency. Organizational performance, on the other hand, is a one-dimensional concept. The empirical relationship is mentioned in the following Fig 2.

**Fig 2:** Hypothetical relationship. https://docs.google.com/document/d/1xej1bG-7xIIvenG5J8oXO5_bThehM8to/edit?usp=sharing&ouid=109167264099591876564&rtpof=true&sd=true.

## 4. Methodology

The research follows a quantitative technique and uses a survey methodology inside a cross-sectional design. It is distinguished by its descriptive and causal nature about its objectives. The inclusion of constructs has been crucial in forming the data collection tool. It is standard practice in behavioral research for researchers to use two or more measurements to evaluate a particular construct or scale [11], achieving precise measurements with a single unit can be difficult. In order to ensure both soundness and consistency in the measurements, the study adheres the recommendation and attempts to use pre-tested constructs from prior empirical research whenever practical [38, 41].

### 4.1. Data and sampling

On the basis of accessibility and convenience, the sample was selected. Considering the significant economic significance of manufacturing sector in China, this study selected both 115 small and medium enterprises of China. The selection of the research sample was deliberate, based on accessibility and convenience. The aim was to select a sample of small and medium-sized enterprises across the country. Thus, enterprises were chosen that could contribute to the research objectives. The majority of these enterprises having number of employees in the range of 20–100. The sample size was determined following Hair’s [27, 28] recommendations. To achieve a statistical significance of 80% and attain an R2 value of 0.25 at a significance level of 95%, considering a total of 4 variables in the model, a minimum of 45 observations [27, 28, 42–45] was deemed necessary. A sample of 115 Chinese SMEs was sought in order to lessen the impact of random factors. The firms in the sample are largely involved in manufacturing and majority of the businesses in the sample were started between the years of 1992 and 2009. The data is collected from senior executives of the firms. A preliminary meeting was arranged with the executives of all of the chosen firms taking part in the study to obtain data. A letter introducing the research was given to them at the meeting. Upon receiving positive responses to the study invitation, the questionnaire was forwarded to the HR representatives of the companies. Approval for the research was obtained from the top management of the participating organizations. The appropriate times for data collection were then established. The data is collected from February 1, 2023 to April 30, 2023. A written consent was gained from respondents prior to fill the survey. The response was received via print form and electronic surveys. The characteristics of respondents are given in the following Table 1.

The article "Unveiling the Nexus: Influence of learning motivation on organizational performance and innovative climate of Chinese firms" was retracted in 2024. Reasons: unreliable data; unreliable results or conclusions; concerns about the data; concerns about the results or conclusions.

**Table 1:** Characteristics of respondents.

Characteristics	Category	Frequency	Percentage
Gender	Male	66	57.39
	Female	49	42.61
Marital Status	Married	78	67.83
	Unmarried	37	32.17
Length of Service	0–5 Years	69	60.0
	6–10 Years	28	24.35
	More than 10 Years	18	15.65
Age	Up to 25 Years	51	44.35
	25–30 Years	48	41.74
	More than 30 Years	16	13.91
Education	High School	32	27.83
	Bachelor	57	49.57
	Master and above	26	22.61
Number of Employees in Firm	Up to 30	56	48.70
	31–60	44	38.26
	More than 60	15	13.04

### 4.2. Measurement

The four factors that make up the notion of organizational learning capability are engaged with the external environment, propensity to risk, and dialogue. The statements for evaluation were created using a seven-point Likert scale, with 1 denoting "completely disagree" and 7 denoting "completely agree". Two components make up the creative performance construct: efficacy, which has seven indicators, and efficiency, which has four indicators. To assess the construct of organizational performance, four indicators were employed, comprising two of financial performance (profitability and return on investment) and two linked to market performance (customer loyalty and sales growth). When financial statement data is either not available or does not allow for precise judgments between organizations, indirect measures of organizational enactment then similar to those were used in earlier studies [14, 35, 46]. The justification for using subjective scales stems from both the unwillingness of businesses to provide accurate performance records and the typical reluctance of managers to divulge objective performance statistics. The Confirmatory Factor Analysis (CFA) was used to analyze the data and evaluate the validity and reliability of the components. The Smart PLS Program was used as the operational tool for the subsequent Structural Equation Modelling (SEM) procedure. The structural model, which follows the methodology described by the study [39, 1, 47–50], illustrates the connections between the variables and quantifies the explained variation. This analytical method was embraced in order to explore the relationships between factors under analysis and verify a model for determining how organizational learning affects innovative performance and how that in turn affects organizational performance. Separate computations were made in order to evaluate the dependability of each construct. PLS-SEM is a popular statistical technique used for analyzing structural relationships between latent variables in empirical research. In summary, smart PLS is used to apply SEM to determine the relationship of considered variables for this study.

The article "Unveiling the Nexus: Influence of learning motivation on organizational performance and innovative climate of Chinese firms" was retracted in 2024. Reasons: unreliable data; unreliable results or conclusions; concerns about the data; concerns about the results or conclusions.

Cronbach’s alpha (CA) is a regularly used dependability method, and values above 0.7 are typically regarded as satisfactory. Hence, alongside Cronbach’s alpha (CA), we also utilized composite reliability (CR) and average variance extracted (AVE). Internal consistency is determined by composite reliability (CR), with values over 0.70 being advised. The reliability measure AVE, on the other hand, shows the percentage of the variance in indicators that can be accounted for by the latent hypothesis and values for AVE greater than 0.5. The discriminant validity indicates the independence of constructs or latent variables from one another, was a crucial factor taken into account while evaluating the models fit [1]. By comparing the associations between the constructs to the square root of the Average Variance Extracted (AVE) for each construct, the Fornell and Larcker [50] criterion was used in the first stage. Each construct’s square root of the AVE must be greater than its correlation with other constructs in order for discriminant validity to be established. These criteria check that item factor loadings are higher on the relevant constructs than on other constructs to support discriminant validity. The t-test values should be greater than or equal to 1.96, were taken into account by the study to determine the significance of the models [1]. Furthermore, the p-value must be lower than 0.05. To evaluate the utility of the constructs in the model, the effect size also known as the Cohen indicator or f2. The effect sizes of 0.02, 0.15, and 0.35 are categorized as small, medium, and big, respectively [41–43]. The study next looked at the results of the structural model and tested the hypotheses after evaluating the goodness-of-fit indicators.

## 5. Estimated results

Table 2 shows the outcomes of calculating coefficients such AVE (Average Variance Extracted), CC (Composite Reliability), and CA (Cronbach’s Alpha).

The article "Unveiling the Nexus: Influence of learning motivation on organizational performance and innovative climate of Chinese firms" was retracted in 2024. Reasons: unreliable data; unreliable results or conclusions; concerns about the data; concerns about the results or conclusions.

**Table 2:** Reliability tests.

Constructs	AVE	CR	CA	R^2^
**Organizational Learning Motivation(OLM)**	**0.429**	**0.844**	**0.809**	**-**
Experimentation(EXP)	0.773	0.982	0.912	0.615
Risk(RSK)	0.721	0.883	0.877	0.654
Interaction(ITR)	0.769	0.904	0.843	0.516
Dialogue(DLG)	0.795	0.805	0.809	0.724
**Innovation Performance(INP)**	**0.842**	**0.961**	**0.925**	**0.528**
Efficiency(EFN)	0.835	0.937	0.866	0.765
Efficacy(EFC)	0.627	0.853	0.866	0.693
**Organizational Performance(ORP)**	**0.764**	**0.993**	**0.915**	**0.696**

AVE, average variance extracted; CA, Cronbach’s alpha; CR, composite reliability

Regarding the AVE values, it’s important to note that merely the second-order paradigm of organizational learning exhibited a value below 0.5, with an AVE of 0.429. However, this particular analysis should be interpreted cautiously, given that the second-order construct comprises all four dimensions of the first order. It’s worth mentioning that an AVE value below 0.5 is not an absolute issue, as some other authors [44] have considered such values acceptable. When examining the Composite Reliability (CR), it is noteworthy that all dimensions scored above 0.70, indicating good internal consistency. Furthermore, looking at the standards of Cronbach’s Alpha (CA), all exceeded 0.7, reinforcing the notion of good reliability. According to the reliability findings, it can be said that the constructions showed sufficient levels of dependability to assessment of the fundamental model. The R-squared (R2) statistic is used to gauge how well the structural model accounts for endogenous variable variation. R2 levels can be characterized as considerable, moderate, or weak, with values close to 0.75, 0.50, and 0.25, respectively. Cohen proposed that R2 = 2% is a minor effect in the social sciences and behavioral disciplines, R2 = 13% is an average effect, and R2 = 26% is a large effect. As can be seen in Table 2, every R^2^ value was greater than 26%, suggesting a significant effect, which is an indication of a good model.

To prove discriminant validity, the study applied Fornell and Larcker’s criteria for discriminant analysis. Through this method, it is determined whether a model’s indicators are unique to one construct or can be distinguished from those of other constructs. The square root of the AVE is greater than the correlations with other latent variables, which is evidence that the model has discriminant validity. Meeting these requirements demonstrates discriminant validity, proving that various measurements relate to various concepts. Discriminant validity was evaluated across all dimensions in accordance with Fornell & Larcker’s criteria. The square root of the AVE was found to be greater than the correlations with other latent variables. In light of these evaluations, it can be said that the model’s constructs show both reliability and validity. The t-test values for each claim were carefully examined using the criterion of 1.96 [1] and p-value > 0.05. There was no need for any revisions at this point because every assertion complied with these requirements. According to Fornell and Larcker’s [50] criterion, Table 3 shows the results of discriminant validity.

The article "Unveiling the Nexus: Influence of learning motivation on organizational performance and innovative climate of Chinese firms" was retracted in 2024. Reasons: unreliable data; unreliable results or conclusions; concerns about the data; concerns about the results or conclusions.

**Table 3:** Discriminant validity.

Dimension	EXP	ITR	RSK	DLG	EFC	EFN	PRF
EXP	**0.820**						
ITR	0.313	**0.759**					
RSK	0.326	0.458	**0.867**				
DLG	0.676	0.416	0.606	**0.880**			
EFC	0.322	0.396	0.522	0.606	**0.818**		
EFN	0.269	0.586	0.638	0.521	0.699	**0.805**	
PRF	0.409	0.340	0.666	0.402	0.695	0.622	**0.685**

Then, a Q2 (predictive validity, also known as the Stone-Geisser indicator) and f2 (effect size, also known as the Cohen indicator) analysis was carried out as shown in Table 4.

**Table 4:** Predictive validity and size effect.

Constructs	(*Q*^2^)	(*f*^2^)
Dimensions of First Order		
EXP	0.380	0.620
RSK	0.385	0.483
ITR	0.428	0.476
DLG	0.469	0.564
EFN	0.617	0.660
EFC	0.546	0.475
ORP	0.362	0.691
Dimensions of Second Order		
OLM	0.000	0.352
INP	0.226	0.460

The goodness of fit is traditionally intended to assess the overall quality of a model. After findings the goodness of fitness, we can estimate the structural equation model and findings are shown in Fig 1. The choice of Partial Least Squares Structural Equation Modeling (PLS-SEM) as the analytical method can be justified on several grounds. PLS-SEM is particularly suitable for models with complex relationships and multiple latent variables, as is the case in this study. It allows for the estimation of both the measurement model (relationships between observed and latent variables) and the structural model (relationships between latent variables) simultaneously, making it ideal for studying the interplay between learning motivation, organizational performance, and the innovative climate. PLS-SEM is known for its ability to handle small sample sizes effectively, which is often the case in organizational research, especially in the context of Chinese firms where data collection can be challenging. PLS-SEM requires a smaller sample size compared to other SEM approaches, making it a practical choice for this study. PLS-SEM is well-suited for prediction-oriented research, where the focus is on understanding and predicting the relationships between variables rather than testing complex causal relationships. In this study, the aim is to predict how learning motivation influences organizational performance and the innovative climate, making PLS-SEM a suitable choice. PLS-SEM offers greater flexibility in model specification compared to other SEM approaches. It allows researchers to include both formative and reflective constructs in the model, which is beneficial when studying complex phenomena such as learning motivation and organizational outcomes. This approach accommodates differences in measurement models and structural relationships across different cultural contexts, allowing for a more nuanced analysis of the impact of learning motivation in Chinese firms. PLS-SEM is a robust analytical method that aligns well with the objectives and requirements of the study, making it a suitable choice for analyzing the impact of learning motivation on organizational performance and the innovative climate of Chinese firms. While PLS-SEM may be considered less robust for confirmatory analysis compared to covariance-based SEM, its ability to handle complex models, small sample sizes, and prediction-oriented research makes it well-suited for exploratory and theory-building studies. The Fig 3 shows the empirical analysis of structural equation model.

The article "Unveiling the Nexus: Influence of learning motivation on organizational performance and innovative climate of Chinese firms" was retracted in 2024. Reasons: unreliable data; unreliable results or conclusions; concerns about the data; concerns about the results or conclusions.

**Fig 3:** Structural equation model. https://docs.google.com/document/d/1ngt-s12u2QFTq8WTmhegLS9tSKtGd3no/edit?usp=sharing&ouid=109167264099591876564&rtpof=true&sd=true.

The results suggest that the relationships proposed within the second-order construct of organizational learning capability and its first-order variables, namely experimentation, interaction with the external environment, propensity to risk, and dialogue hold validity within the context of organizational learning capability. Organizational learning is the cooperative creation of new shared meanings through communication, equitable involvement, and a readiness to accept divergent opinions. Shared experiences and unrestricted access to information define it. In these situations, productive conversations are essential to the organizational learning process. Notably, "Dialogue" had the greatest impact on the organizational learning capabilities of all the dimensions. By establishing routines for communication among various groups or levels of the hierarchy, bureaucratic processes are reduced, which promotes greater consistency and innovation. This is because people come to share a common thought process and have a better awareness of the issues and objectives of the organization [45, 51]. The findings also point to the prevalence of work teams, which are frequently made up of individuals from other industries. The exchange of open knowledge inside these work teams may produce new results [46, 52]. This demonstrates how information sharing and cross-functional cooperation may help firms to innovate. Notably, the efficacy dimension exhibited the highest factor loading, indicating a strong association with innovations introduced in the market. This suggests that the effectiveness of innovation efforts, particularly in terms of introducing new products to the market, played an essential role in the overall assessment of innovative performance. It appears that the small and medium-sized companies are primarily focused on staying competitive in the market by continuously innovating their product offerings to align with the evolving demands of a sector that consistently seeks novelty. These companies operate in an industry marked by a diverse range of products with exceedingly short lifecycles, largely dependent on ever-changing fashion trends. The cost and duration of innovative project have a significant impact on the efficiency dimension, which has a significant value. This shows that these businesses place a high priority on time and cost control while creating creative projects. Given that these businesses often face competition from larger corporations, it’s apparent that they prioritize cost-effectiveness to remain competitive. Additionally, the rapid changes in fashion trends are another factor contributing to this focus on efficiency. In an industry characterized by fast-changing trends, organizations need to develop products that can quickly adapt to these shifts and endure in the marketplace for short-term periods. Table 5 displays the results of the hypotheses testing in the study, which further elucidate these dynamics.

The article "Unveiling the Nexus: Influence of learning motivation on organizational performance and innovative climate of Chinese firms" was retracted in 2024. Reasons: unreliable data; unreliable results or conclusions; concerns about the data; concerns about the results or conclusions.

**Table 5:** Hypothesis testing.

Structural Path	Path Coefficients	SE	T values	P-Value	Results
OLM → INP	0.420	0.049	8.571	0.000	Supported
INP → ORP	0.462	0.062	7.451	0.000	Supported
OLM → ORP	0.358	0.025	6.882	0.003	Supported

Table 5 demonstrates a positive and significant correlation between organizational learning motivation and innovation performance. According to the standards set by the study [40], the T-values which exceeded 1.96, indicates that the coefficients are resilient.

## 6. Discussion

These findings of the study confirm the Hypothesis 1, according to which firms perform more innovatively when organizational learning is made easier. Earlier studies [35, 47, 53–55] highlight the crucial role of learning in helping firms to attain agility and flexibility in the innovation process. In fact, a firm with excellent knowledge integration and acquisition skills is more likely to succeed in both product and process innovation, leading to better results in the creation of new goods. A company is likely to do well in terms of product and process innovation if it can successfully incorporate new information into its current knowledge base through a variety of techniques. Simply put, an organization’s performance in innovation is likely to be more impressive the higher its capacity for organizational learning. Organizational learning motivation encourages employees to seek out new knowledge and skills, which can stimulate creativity and innovative thinking. When employees are motivated to learn and explore new ideas, they are more likely to come up with innovative solutions to problems. A strong learning culture within an organization promotes knowledge sharing among employees. When employees are motivated to learn from each other, they are more likely to share their knowledge and experiences, leading to a more innovative and collaborative work environment. It also helps employees to develop a mindset that is open to change and new ways of doing things. This adaptability is crucial for innovation, as it allows organizations to respond effectively to changing market conditions and emerging trends [47]. Learning motivation encourages employees to continuously improve their skills and knowledge. This focus on continuous improvement can lead to incremental innovations that enhance organizational performance over time. A culture of learning and experimentation encourages employees to take risks and try out new ideas. This willingness to experiment is essential for innovation, as it allows organizations to test new concepts and approaches without fear of failure [32]. Organizations that prioritize learning and development tend to have higher levels of employee engagement and satisfaction [42]. Engaged and satisfied employees are more likely to be innovative and contribute positively to organizational performance. Overall, the positive relationship between organizational learning motivation and innovative performance highlights the importance of creating a learning culture within an organization [31]. By fostering a culture that values learning, organizations can drive innovation and improve their overall performance.

The article "Unveiling the Nexus: Influence of learning motivation on organizational performance and innovative climate of Chinese firms" was retracted in 2024. Reasons: unreliable data; unreliable results or conclusions; concerns about the data; concerns about the results or conclusions.

The findings for Hypothesis 2, states that innovation performance influences organizational performance with a favorable and significant relationship. These results underline the standing of innovation in improving organizational enactment and lend credence to the view that innovation is a major factor in an organization’s long-term success. Many studies have looked at the connection between innovation and performance, and they regularly show that there is an advantageous relationship. For example, studies [9, 30, 56–59] have demonstrated that innovation contributes to increased organizational performance, highlighting the importance of innovation in achieving positive organizational outcomes. The aspiration of firms to improve their organizational performance and obtain a reasonable edge drives the adoption of innovations [60–62]. Companies recognize that the extent to which they prioritize innovation corresponds with their ability to secure additional competitive advantages and expand their market share. Innovations serve as a pivotal factor for SMEs to establish a strong market status and, consequently, to bolster their marketplace presence and influence [31, 63–65]. SMEs that excel in organizational learning are better equipped to discern market events and trends. Consequently, these learning organizations tend to be more adaptable and swift in their responses to new challenges compared to their competitors. This agility allows them to maintain competitive advantages over the long term [18, 66–68].

It can be argued that innovation performance directly contributes to a company’s competitive advantage. Organizations that consistently innovate are able to differentiate themselves from competitors, attract customers, and capture market share. This can lead to increased revenue and profitability, which are key components of organizational performance [46]. Innovation often leads to improvements in productivity and efficiency. New technologies, processes, or products developed through innovation can help organizations streamline their operations, reduce costs, and increase output. This can result in higher levels of organizational performance as measured by metrics such as return on investment (ROI) and operational efficiency [64]. Innovation can open up new markets and business opportunities for organizations. By developing new products or services that meet the needs of previously untapped customer segments, organizations can expand their market reach and grow their business. This can have a positive impact on organizational performance by increasing market share and revenue [35]. Organizations that are known for innovation often enjoy a strong reputation in the marketplace. This can lead to increased customer loyalty, positive brand perception, and a competitive edge. A strong reputation can contribute to organizational performance by attracting top talent, fostering partnerships, and enhancing shareholder value [49]. Innovation can help organizations manage risk by diversifying their product or service offerings and revenue streams. By continually innovating, organizations can reduce their dependence on a single product or market, making them more resilient to economic downturns or industry disruptions. Organizations that prioritize innovation are more likely to achieve sustainable growth and success in the long run.

The article "Unveiling the Nexus: Influence of learning motivation on organizational performance and innovative climate of Chinese firms" was retracted in 2024. Reasons: unreliable data; unreliable results or conclusions; concerns about the data; concerns about the results or conclusions.

There is a positive correlation between the learning motivation of organizations and their performance. As a result, the findings also support Hypothesis 3, which states that organizational learning characteristics have a favorable impact on overall performance of firms. Organizational learning motivation is shown to be correlated with organizational performance [69, 70]. But it is important to preserve in mind that innovation is a proven factor in determining how well a business performs [30, 71]. It is possible to infer that innovation mediates the link between knowledge and organizational performance. In other words, the advantages of organizational learning may be realized through the innovation process, which will ultimately affect organizational performance. To put it another way, organizational learning motivation affects innovation performance, which in turn affects organizational performance [1, 72]. This demonstrates the intricacy of the connections between organizational learning, advancement, and performance, which can differ between and within organizations and in different circumstances. In the long run, learning is necessary for greater performance [43, 73]. As a result, organizational learning is frequently seen as a key component of success within a corporation. Moreover, it is emphasized that the ability to learn faster than one’s rivals might be a source of long-term competitive advantage [27, 31, 74].

The earlier study not only highlights the positive influence of organizational knowledge on performance but also emphasizes the arbitrating role of innovation in this association. Several studies propose that organizational learning equips a company with the capabilities needed to enhance innovation, and that revolution, in turn, has optimistic effect on overall performance [34, 48, 75, 76]. Therefore, organizations that prioritize innovations should also promote organizational learning, as this can help optimize the effect of innovative performance on overall organizational performance. This underscores the interconnectedness of learning, innovation, and organizational success [49–51, 77]. The outcomes of this investigation support the notion that organizational learning capability is essential for fostering creativity. SMEs should therefore emphasize and improve their organizational learning procedures if they want to advance their enactment through innovation [52, 78]. This finding is especially important for smaller businesses and those operating in extremely dynamic and chaotic situations. For long-term success and competitiveness in such environments, the capacity to learn, adapt, and innovate becomes even more essential. The performance of the surveyed organizations was positively impacted by the elements that support organizational learning [53]. It is obvious that having a strong capacity for learning is essential for innovation and, in turn, enhances organizational success. These findings offer valuable insights to managers, particularly within the context of SMEs, by emphasizing the importance of incorporating displays of organizational learning ability into their supervision tools. This enables the effective implementation of conditions that promote learning within organizations, ultimately enhancing their innovative capacity and overall performance [54, 79, 80].

The article "Unveiling the Nexus: Influence of learning motivation on organizational performance and innovative climate of Chinese firms" was retracted in 2024. Reasons: unreliable data; unreliable results or conclusions; concerns about the data; concerns about the results or conclusions.

## 7. Implications

### 7.1. Theoretical implications

Theoretical implications of this research contribute to several key areas of social learning theory, goal setting theory, and organizational theory. This research deepens the understanding of these theories explaining the relationship between learning motivation and organizational performance within the context of firms. It provides theoretical insights into how individual-level factors, such as motivation, influence broader organizational outcomes, shedding light on the mechanisms through which employee behaviors and attitudes impact organizational effectiveness. The research has implications for human resource management practices related to employee motivation, training, and development. By identifying the factors that drive learning motivation and their impact on performance and innovative climate, organizations can develop more effective strategies for recruiting, retaining, and motivating employees, as well as designing training and development programs that align with organizational goals. The research also contributes to the literature on innovation management by highlighting the importance of learning motivation in fostering an innovative climate within firms. The research also extends theoretical frameworks of organizational learning by examining how learning motivation influences organizational performance and innovative climate. It contributes to our understanding of the dynamics of learning within organizations, including the mechanisms through which learning motivation drives knowledge acquisition, sharing, and application, as well as the factors that facilitate or inhibit a culture of continuous learning and improvement.

### 7.2. Practical implications

The findings of this study provide some useful insights for managers of SMEs. It underlines the significance of concentrating on the elements that support organizational learning since these elements both directly and indirectly affect both innovation and organizational success. Within the company, it is indispensable to have a broad-mindedness for vagueness, hesitation, and mistakes. The results emphasize how important it is to listen to fresh ideas and comments from staff members. Innovation is a crucial requirement for survival and ongoing success in the cutthroat atmosphere. Therefore, in order to succeed in this competitive corporate environment, managers need actively promote a culture of learning and innovation. The "Dialogue" component stands out as having the greatest influence on organizational learning. Improving communication is essential for improving knowledge sharing inside the organization. By using cross-functional work teams, managers may formally establish procedures to encourage the exchange of best practices between departments and among employees. Additionally, managers can support original and imaginative methods for problem solving. Promoting the acquisition of new information is vital for SMEs. This may be done by encouraging staff members to routinely attend fairs and exhibitions by highlighting the benefits of networking, learning about new technologies and trends, and gaining insights into competitors, which will help them to acquire fresh perspectives and encounter new things outside of the organization. SMEs can provide financial support for registration fees, travel, and accommodation to make it easier for staff to attend these events. Encourage staff who attend these events to share their insights and learning with the rest of the team through presentations, reports, or informal discussions. Attending fairs and exhibitions exposes staff to new products, technologies, and trends in the industry, which can stimulate innovation and new ideas within the organization. These events provide opportunities to network with industry peers, potential partners, and suppliers, which can lead to collaborations and business opportunities. Attending these events can contribute to the professional development of staff, enhancing their knowledge and skills, which can benefit the organization. By staying informed about the latest industry developments, SMEs can gain a competitive edge over rivals who may not be as well-informed. Incorporating these techniques and fostering a culture of open communication and information sharing may promote organizational learning and, as a result, lead to increased innovation and performance in SMEs.

The article "Unveiling the Nexus: Influence of learning motivation on organizational performance and innovative climate of Chinese firms" was retracted in 2024. Reasons: unreliable data; unreliable results or conclusions; concerns about the data; concerns about the results or conclusions.

### 7.3. Limitations and future research

Despite the study’s strict adherence to the recommended methodology, there are a few limitations that should be considered while analyzing the results. The research focused exclusively on SMEs located in China, potentially limiting the generalizability of the findings. Relying on a single respondent as the primary data source may introduce bias, and employing a social desirability scale could provide deeper insights into responses. It is advised that future studies should examine contingency elements that affect organizational effectiveness and creativity. Studies might also look on the differences in innovation across the industrial and service industries. Additionally, longitudinal research should be taken into consideration in order to evaluate how organizational performance and learning capabilities change over time. The relationship between learning capacity and performance over time may be supported by longitudinal data, and one component of this relationship is an examination of the relationships between financial and non-financial performances.

## 8. Conclusion

The purpose of this study was to explore the relation among organizational learning motivation, overall organizational performance and innovative performance of SMEs. The findings demonstrate that organizational learning motivation influence the organizational performance in context of innovations. The link between organizational learning and innovation performance demonstrates that learning is the basis for the creation of new products and processes since these innovations are impacted by factors that foster the learning process inside these SMEs. This highlights how essential organizational learning is to encouraging innovation, which may therefore have a positive impact on a company’s success.

The results of the study provide insightful theoretical information and may inspire more investigation in the area. The work advances the evaluation of learning capacities by showing important theoretical implications that are not readily observable. Additionally, by examining the connections between the organizational learning, innovations, and performance within a single model and using units that have been verified in global contexts, this study is an addition to the body of literature. This paper offers empirical support for these linkages, demonstrating their significance and beneficial nature, particularly for SMEs in China. This is especially significant in the empirical research of this field, which makes this study an important addition to our knowledge of organizational dynamics and performance in such settings.

The fast paced nature of the fashion sector supports an innovative culture. The ongoing testing of novel strategies for more effective management and product development is encouraged by this culture. It forces businesses to embrace this cutting-edge viewpoint, which increases their openness to implementing novel practices and technology. The industry’s dedication to innovation is driven by its need to remain competitive and adaptable in the ever-changing fashion landscape.

The article "Unveiling the Nexus: Influence of learning motivation on organizational performance and innovative climate of Chinese firms" was retracted in 2024. Reasons: unreliable data; unreliable results or conclusions; concerns about the data; concerns about the results or conclusions.

## Supporting information

S1 Data (XLSX)
